The article "Analyzing Intention to Purchase Brand Extension via Brand Attribute Associations: The Mediating and Moderating Role of Emotional Consumer-Brand Relationship and Brand Commitment" was retracted in 2025. Reasons: unreliable results or conclusions; a conflict of interest; concerns about the peer review; concerns about the citations.

# Analyzing Intention to Purchase Brand Extension via Brand Attribute Associations: The Mediating and Moderating Role of Emotional Consumer-Brand Relationship and Brand Commitment

**DOI:** 10.3389/fpsyg.2022.884673

**Published:** 2022-07-15

**Authors:** Weijun Bian, Gong Yan

**Affiliations:** ^1^School of Literature and Business, Xi’an Siyuan University, Xi’an, China; ^2^School of Urban Construction, Xi’an Siyuan University, Xi’an, China

**Keywords:** brand extension, brand attribute, luxury brand, commitment, emotional consumer-brand relationship, purchase intention

## Abstract

The aim of this study is to investigate the drivers of brand extension attributes and its impact on intention to purchase brand extensions mediated by emotional consumer-brand relationship (ECBR). Data was collected from Chinese university students with the help of questionnaire. Structure equation modeling was applied with the help of AMOS to analyze collected data. Results depict that brand attribute association has significant impact on intention to purchase luxury brands extension. Results further explain that emotional consumer-brand relationship mediates the relationship between brand attribute associations and purchase intention of brand extensions. Furthermore, results indicate that brand commitment moderates the relationship between brand attribute associations, emotional consumer-brand relationship and intention to purchase brand extensions. This study provides an intensive knowledge of the association that exists between the intent to buy luxury brands’ extension and ECBR. This study focuses on the heart versus mind distinction, which is integral to the research on the relationship between consumers and brands. This study provides useful insights to brand managers to use strategies that enhance the bond between emotional and cognitive factors customers associate with a particular brand. Luxury brand managers ought to balance emotionality and rationality to create and capitalize on unique associations with customers.

## Introduction

Brand extension refers using a brand’s name to facilitate market penetration for a new product and this strategy is used in promoting luxury brands (Zhu et al., 2021). Already a lot of luxurious fashion brands enjoy brand extension across various traditional luxurious market segments like jewelry, accessories, and perfumes; there are also extension possibilities when it comes to the non-traditional segments like technology, accommodation, food, and alcohol. Even though a parent brand name presents a chance for brand extension success, the brand extension also has its fair share of limitations (Gelb and Friedman, 2021). Brand dilution emanates from overextension which contributes immensely to brands losing the special aura or brand promise to the potential market and subsequently reducing their market share. For that reason, it is crucial to determine the determinants that specifically affect the success of a particular luxury brand extension. There has been little study on the drivers of successful luxury brand extensions. The studies on non-luxury brand extensions cannot be used in the luxury brand category hence the need to carry out a separate study on luxury brands (Jamil et al., 2021a; Ma et al., 2021).

According to Knoerzer and Millemann (2021), both relational and cognitive factors play a significant role when it comes to consumer decisions. Tsai et al. (2020) stated that cognitive roots drive consumer emotions (Gul et al., 2021a). When consumers retain brand attributes in their minds, it leads to the consumer-brand association. Consumers always tend to create salient schemas associated with the brand in their mind, thus developing an emotional bond with that brand. Global consumer expenditure growth also challenges organizations to create productive brand associations; thus, it is valuable to create and improve the emotional attachment between customers and luxury brands through taking advantage of cognitive aspects like brand relationships which consumers have imprinted in their minds (Dewani et al., 2021; Gul et al., 2021b). It will also be beneficial to determine whether marketers can get desired results like encouraging consumers to purchase luxury brand extensions through capitalizing on the interplay of these mechanisms. Zhong et al. (2021) discussed that despite this, there appears to be a paucity of research that investigates the influence of cognitive and relational elements (in addition to expected synergies) on brand expansions.

Past studies on the discussed issues have several empirical and conceptual limitations. For instance, Prados-Pena and Del Barrio-García (2021) focused on affective commitment only. Gelb and Friedman (2021) and Hultman et al. (2021) conceptualization about customer-brand association focused on hedonic values and emotional attachment. Zhu et al. (2021) focused on brand elicited effects, that is, feelings experienced by consumers when coming across a brand are different from the emotional attachment between the brand and consumer. Besides, most studies have always put more emphasis on brand quality when it comes to conceptualizing cognitive factors. Other studies did not have generalizability because of the specific assumptions which, may have affected how the findings were interpreted. Take, for instance, Ahn et al. (2018), who argued that emotions tend to be more impacting than attitudes when predicting how consumers will react to luxury brand extensions. However, this only happens when a consumer expects a moderate or high-level fit between brand extension and parent brand. According to del Barrio-García and Prados-Peña (2019), consumers’ judgments on brand extensions are enhanced by strong brand association quality, however only in low and moderate commitment extensions. These limitations have prompted the current study to develop and test the empirical model suitable for examining the importance of emotional consumer-brand relationships (E-CBRs) and brand attribute relationships in determining the intent of a luxury brand extension. ECBR is referred to as an emotional attachment that consumers develop as time goes by with their preferred brands. In addition, this study examines the impact caused by brand commitment (Jamil et al., 2022).

The current study focuses exclusively on luxury brands’ context, adding to the available knowledge about luxury brand consumption. Luxury brands come with specific characteristics, making them viable for examining all aspects that have been discussed. For instance, luxury brands offer consumers benefits that can be transferred across various product categories. Also, luxury brands come with high hedonic and expressive characteristics. According to Kumar and Kaushik (2020), luxury brands are a blend of cognitive and emotionally laden values like entertainment, experiences, aesthetics, and superior quality. Chinese young consumers have experienced tremendous growth when it comes to interest in leading a luxurious lifestyle and using global luxury brands. So, the research analyses views from young consumers in China to draw various practical and theoretical contributions (Gul et al., 2021c). The findings show that the Chinese luxury brand market now boasts of having a wide variety of global luxury brands. Besides, Chinese consumers have interesting behaviors, like marked impacts of cultural factors, that ate worth studying for a lot of global investors and brands.

## Literature Review and Hypotheses Development

### Consumer Intention to Buy Brand Extensions and Brand Attribute Association

Brand attribute associations are descriptive features used in the characterization of a brand, for instance, its intangible benefits, factors that influence consumption or purchasing of a brand, and an image that resonates well with consumers (Prados-Peña and Del Barrio-García, 2020). This study appreciates the views of Butcher et al. (2019) in describing the conceptualization of brand attributes associations. There are five main dimensions that consumers highly value regarding luxury brands. Among those dimensions (perceived quality, perceived originality, and prestige/elitism/conspicuousness) are associated with non-personal attributes, while the remaining two (perceived extended self and perceived hedonism) are related to personal values. According to Tsai et al. (2020), luxury values are represented by three dimensions (hedonism, distinction, and elitism/prestige). When it comes to luxury brands, consumers usually perceive materialism and hedonism as individual values, conspicuousness, and prestige to be social values, uniqueness, and quality as functional values (Awan et al., 2021a).

Liang and Fu (2021) have confirmed that intention to purchase brand extensions is a result of associations with brand attributes. For example, suppose a consumer comes across new brand extensions. In that case, their evaluation of the brand extensions is based on the parent brands’ attributes and the knowledge they currently have concerning that product category (Kumar and Kaushik, 2020). Besides, theoretical support on how the purchase intention of a brand extension is influenced by these dimensions. For instance, Youn and Dodoo (2021) confirm that the brand image is likely to influence the perceived quality of the brand even before making a purchase. So, these dimensions influence how a consumer will evaluate a brand extension (Awan et al., 2021b; Ma et al., 2021). Hedonic attributes from the parent brands also affect how consumers perceive a brand and promote the development of feelings by a consumer toward a brand (Tseng et al., 2022). These attributes can be used on new products irrespective of the categories they fall in. Brand prestige suggests that the likeability or relatability of a parent brand affects how brand extensions are evaluated (Giovanis and Athanasopoulou, 2018; Jamil et al., 2021b). Researchers have also pointed out that the values provided by a brand (functional and prestige values) influence how consumers will react to brand extensions. A parent brand with prestigious values might negatively impact consumers’ purchasing decisions in the event of a brand extension by providing highly perceived quality (Nandy and Sondhi, 2020). Finally, brand uniqueness refers to extrinsic or inter-personal advantages brought by brand consumption and is important when customers tell other potential customers about their first-hand experience regarding a particular brand. Brand extensions can enjoy such benefits (Awan et al., 2021c; Zhong et al., 2021).

There are a number of major conceptual and empirical constraints in the existing research that examines consumer-brand relationships as a factor in evaluating brand expansions. These limitations affect the study in both a conceptual and an empirical way (Tseng et al., 2021). Even though a lot of research has been done on the impact of intention to purchase a brand extension. But studies regarding luxury brands confirm that consumers depend on the attributes of the parent grand in creating perceived quality of brand extensions (Gaber et al., 2021; Mohsin and Ivascu, 2022). Consumers often use those attributes to determine the benefits they stand to gain after purchasing brand extensions. Positive attributes of the parent brand will enable consumers to positively evaluate the brand extension (Mohsin et al., 2021). The quality of a brand’s connection to its consumers and the degree to which consumers feel that the brand is a good match for them both have separate and distinct impacts on how consumers feel about the growth of the brand. However, their findings only revealed a substantial influence on behavioral reactions to brand growth, not on views toward the expansion of the company. This is because opinions are more subjective. Dewani et al. (2021) found that only extensions with moderate to low fit had a favorable influence on consumer perceptions of good brand connection quality. This meant that only extensions with a moderate to low fit had a positive impact. In other research, it was investigated how customers’ impressions of the parent firms changed as a result of the introduction of new brands. According to Gorlier and Michel (2020), unique, prestige, and hedonic values positively impact how consumers perceive brand extensions. Therefore, we proposed following hypothesis:

H1a: Emotional consumer-brand relationship (ECBR) impacts consumer intentions to purchase a brand extension and brand attribute associations.

### The Moderating Role of Brand Commitment

A strong sense of psychological attachment toward an object is regarded as a commitment (Das et al., 2019). It is an enhanced urge to have a certain attitude, and it binds or pledges the person to a particular behavior. Various forces around the individual (culture and social network) and consumer experience are the drivers of commitment (Piehler, 2018; Liu et al., 2019). Affective attachments and emotions influence a particular object. So, commitment comes with positive feelings and customer partiality (Abid et al., 2020).

According to Tong et al. (2018), it is possible to transfer an emotional attachment from one object to another. An individual with a deep attachment to a certain object tends to stay committed to preserving the relationship with it. Besides, Kumagai and Nagasawa (2021) also confirmed that high attachment to brand extensions occurs at the high levels of fit. So, the effect will only be transferred depending on the emotional attachment toward the brand extension and its similarity to the main brand (Liu et al., 2017; Ou et al., 2020). In an instance where the brand extensions display high perceived quality, they can easily be regarded to have similar features to the parent brand (Gul et al., 2021d). So, the effect is transferred with an enhanced commitment condition. Therefore, we proposed following hypothesis:

H1b: Brand attribute associations significantly affect intention to emotional consumer relationship (E-CBR).

### The Mediating Role of Consumer-Brand Relationship

A substantial degree of synergy exists between E-CBR and brand attribute associations while influencing the intention to buy brand extensions (Kaufmann et al., 2019). Gupta et al. (2021) confirm that emotions facilitate brand-associated information when making purchase decisions, mostly if unique, conspicuous, and hedonic attributes affect the decision. Besides, the relationship between a consumer and a brand often becomes a conduit linking purchase decisions and the brand extensions’ cognitive factors (perceived quality or brand image). One can determine whether brand relationships are mediating by putting into consideration emotions resulting from a consumer’s bond with a particular brand that usually affect the consumer’s purchasing decisions (Pourazad et al., 2019; Naseem et al., 2021).

Still, these works have theoretical and conceptual frameworks that should be subjected to additional empirical analysis. Even though, according to Loureiro and Sarmento (2019), emotional reactions are more effective than perceived fit and attitudes when predicting how a consumer will react to the brand extension. This confirmation is only viable for moderate and high levels of brand extensions and parent brands. Besides, Hayes et al. (2020) framework put more emphasis on a single aspect of brand relationship development (hedonic benefits from parent brands). Also, the works of Khatoon and Rehman (2021) on perceptual factors dwelt on the quality of brand portfolio and parent brand breadth. Furthermore, Gaber et al. (2021) used the dyadic approach, appraised brand relationship, hence hindering conclusions generalizability. Therefore, we proposed following hypothesis:

H2: Brand attribute has a significant influence on intention to purchase a brand extension.

### Brand Attributes and Intention to the Emotional Consumer-Brand Relationship

Past studies acknowledge the significance of the interaction between relational and cognitive factors and how they affect customer decisions (Schmuck et al., 2018). Successful brands establish a productive relationship with consumers through providing an exceptional combination of product benefits and perceptual brands. According to Yazdanparast et al. (2016), brand image assists in creating brand relationships in case consumers consider self-image to be consistent with the perceived quality. Consumers use the unique intangible benefits of a brand to evaluate a brand or develop feelings toward it (F. Hu and Trivedi, 2020).

According to the Theory of Optimal Distinctiveness (Hornsey and Hogg, 1999), individuals tend to join moderately distinct and inclusive groups to fill different or simply fulfill the demand for inclusion (Liu et al., 2021). Besides, consumers always display their identities by associating with prestigious brands to gain status, respect, and exclusivity. According to Social Identity Theory, an individual embodies the attributes of social identity, which assist them in realizing positive, aspirational targets. As social identities, brands have prestigious attributes that attract consumers, making them develop attachments with the brand (Liu et al., 2020). According to Sultan and Wong (2019), congruency between a consumer’s ideal self and the brand impacts brand attachment positively. Hayes et al. (2021) also suggest that hedonic and symbolic benefits can cause brand attachment. As a result, this study proposes these hypotheses:

H3: Brand commitment mitigates the relationship between intentions to purchase a brand extension and the emotional consumer-brand relationship.
H4: Brand commitment mitigate the relationship between intention to purchase brand extension ad brand attribute associations (see Figure 1 for all relationships).

**FIGURE 1:** Conceptual framework.

### Research Methodology

Data was collected from respondents using a self-administered questionnaire. Before the final analysis a pilot study was conducted with first thirty and last thirty questionnaires. After the results of pilot study two experts of the marketing field reviewed the questionnaire items and the responses of the respondents and they suggested some minor revisions to improve the quality of the instrument. Non-probability convenience sampling technique was applied to collect data from university students situated in Beijing the capital of PR China. Though convenience sampling may constitute a generalizability issue, researchers suggested that young samples are more accurate and knowledgeable about fashion products. This study follows the suggested sample size criterion of Kline (2015). According to him ten responses for an item are sufficient. Our study used twenty-five items and the minimum suggested sample should be two hundred and fifty. Keeping in view the reliability and validity we collected data from three hundred and twenty-five Chinese students who are studying in different universities in the territory of capital city Beijing.

### Questionnaire and Measurement

The study used items established from prior research to confirm the reliability and validity of the measures. All items are evaluated through five-point Likert-type scales where “1” (strongly disagree), “3” (neutral), and “5” (strongly agree). Intention to purchase brand extension was measured with three items adopted which were adopted from prior study of Taylor and Baker (1994). Brand attribute association was evaluated with eleven items and these items were previously used by Hwang and Hyun (2012). Emotional Consumer-Brand Relationship (E-CBR) was used as mediating variable and this was determined with the help of eight items which already were used by Carroll and Ahuvia (2006) and Batra et al. (2012). To check moderating effect of brand commitment we used three items and these items were formerly used by Albert et al. (2013) in their study.

### Demographic Profile of the Respondents

The demographic analysis results showed that 59% of the respondents were male, and 41% were female; participation in both the sample assures the inclusion of genders in the dataset. About 35% of the respondents were aged between 18 and 25 years, followed by 40% aged between 26 and 35 years, and the rest of 25% were above the age of 35 years. Respondents were well-educated, with about 40% were graduation students, and about 45% of respondents were post-graduate students.

## Study Results

The SEM approach has been extensively employed because it can illustrate robust regression associations in a single model and test (Kline, 2015). It is also applicable and rational to determine associations and mediation effects. Therefore, this research employed SEM to assess the proposed hypotheses of the research model. This study utilizes analysis of moment structures (AMOS) to assess and evaluate the structural model based on standardized scale data. CFA was implemented to examine the validity and reliability of the constructs. Data analysis was carried out using statistical package AMOS version 24. In contrast, a bootstrapping technique was utilized to test the significance of the research hypotheses.

### Measurement Model

A confirmatory factor analysis with AMOS 24.0 software on 260 returned survey data was conducted. According to the Structural Equation Model (SEM) index suggested by Bagozzi and Yi (1988), the fit indices of the model are satisfactory (CMIN/DF = 2.229, RMSEA = 0.069; GFI = 0.845; SRMR = 0.050, AGFI = 0.81; CFI = 0.92; TLI = 0.909), suggesting that The CFA findings are an excellent fit to the data (see Figure 2). The detailed findings for the measurement model and cut-off criteria are shown in Table 1.

**FIGURE 2:** Model fit measures.

**TABLE 1:** Model fit measures.

Index	Measurement model	Structural model	Cut-off criteria	Benchmark	Conclusion
**Absolute fit measures**					
CMIN/DF	2.229	2.366	<5.0		Appropriate
RMSEA	0.069	0.073	<0.08	MacCallum et al., 1996	Appropriate
SRMR	0.050	0.051	<0.08	Byrne, 2013	Appropriate
GFI	0.845	0.857	>0.80	Hu and Bentler, 1995	Appropriate
**Incremental fit measures**					
CFI	0.920	0.923	>0.90	Bentler, 1990	Appropriate
AGFI	0.810	0.821	>0.80	Bentler and Weeks, 1980	Appropriate
TLI	0.909	0.913	>0.75	Sivo et al., 2006	Appropriate

Next, we assessed the efficiency of the design measures by measuring the individual Cronbach alpha Ca coefficient, with the resulting estimates varying from 0.832 to 0.935, all of which were higher than the recommended standard of 0.7 (Nunnally, 1994). A CFA was then carried out to test the cumulative measurement model to ascertain the convergent and discriminant validity. Following the guideline of Hair et al. (2016), this research examines the convergent validity through factor loading, average variance extracted (AVE), and composite reliability (CR). The factor loadings of the items range from 0.618 to 0.841 (all larger than 0.6). The CR values are greater than 0.7, and they range from 0.833 to 0.934. AVE values vary from 0.545 to 0.685, all of which are greater than 0.5. All the measures demonstrated sufficient convergent validity, as seen in Table 2.

**TABLE 2:** Confirmatory factor analysis results.

Items	Loadings	Estimate	S.E.	C.R.	CA	CR	AVE	MSV	MaxR(H)
Brand attribute associations					0.935	0.934	0.545	0.121	0.939
BAA3	0.759***	1.094	0.097	11.265					
BAA4	0.841***	1.290	0.104	12.356					
BAA5	0.767***	1.109	0.097	11.382					
BAA6	0.758***	1.049	0.093	11.261					
BAA8	0.759***	1.231	0.109	11.270					
BAA11	0.785***	1.231	0.106	11.616					
BAA12	0.801***	1.240	0.105	11.836					
Emotional consumer Brand relationship					0.904	0.901	0.568	0.404	0.911
ECBR2	0.837***	1.474	0.139	10.610					
ECBR3	0.820***	1.382	0.132	10.466					
ECBR4	0.815***	1.432	0.137	10.422					
ECBR5	0.737***	1.427	0.147	9.7100					
ECBR6	0.711***	1.286	0.136	9.4420					
ECBR7	0.712***	1.303	0.138	9.4570					
Intention to purchase Brand extension					0.866	0.867	0.685	0.088	0.872
IPB1	0.809***	1							
IPB2	0.869***	1.101	0.078	14.190					
IPB3	0.804***	1.019	0.075	13.548					
Brand commitment					0.832	0.833	0.625	0.404	0.841
BC1	0.839***	1							
BC2	0.804***	0.952	0.073	13.106					
BC3	0.724***	0.838	0.071	11.876					

Significance of estimates at ***p < 0.001 level; Cα ≥ 0.7; CR ≥ 0.7; AVE ≥ 0.5.

The two methods are included to validate the proposed model’s discriminant validity, namely the Fornell-Larcker criteria and heterotrait-monotrait (HTMT) ratios (Hair et al., 2016). According to the Fornell and Larcker (1981) criterion, after taking the square root of the AVE of each variable, if the upper side of the first value of each column is significantly higher, it demonstrates the confirmation of discriminant validity (Fornell and Larcker, 1981; Hair et al., 2016). Table 3 indicates that discriminant validity is confirmed based on the Fornell-Larcker criteria since the top value of the association of measures is maximum in each column. According to the HTMT ratios criteria, the values of the HTMT ratios must be <0.85; but, values up to 0.90 are appropriate. The Table 3 demonstrates that all HTMT ratios are <0.90, which suggests that the current research model’s discriminant validity has been confirmed.

**TABLE 3:** Discriminant validity.

Fornell–Larcker criterion					Heterotrait–monotrait (HTMT) ratios				
	BAA	ECBR	IPB	BC		BAA	ECBR	IPB	BC
BAA	0.738				BAA				
ECBR	0.250	0.754			ECBR	0.249			
IPB	0.297	0.266	0.828		IPB	0.297	0.274		
BC	0.348	0.636	0.210	0.790	BC	0.339	0.650	0.209	

*BAA, brand attribute associations; ECBR, emotional consumer-brand relationship; BC, brand commitment; IPB, intention to purchase brand extension.*

### Structural Model Results

We used SEM with maximum likelihood estimation procedures to test the proposal hypotheses. To measure the degree fit of the structural model we evaluated the following indicators: absolute fit measures including Chi-square/df (CMIN/df), goodness of fit index (GFI), root mean square error of approximation (RMSEA) and root mean square residual (RMR), Standardized Root Mean Square Residual (SRMR); incremental fit measures including, comparative fit index (CFI), adjusted goodness of fit index (AGFI), Tucker–Lewis coefficient (TLI). Table 1 shows that the fit indices of the model are satisfactory (CMIN/DF = 2.366, RMSEA = 0.073; GFI = 0.857; SRMR = 0.051, CFI = 0.923; AGFI = 0.821; TLI = 0.913), suggesting that the relationships among latent constructs fits the data. The direct, indirect and total effects are analyzed and shown to clarify the relationship among the factors (Usman Shehzad et al., 2022). The results of the hypotheses testing of the structural relationship among the latent constructs in the proposal model are shown in Figure 3 and Tables 4, 5.

**FIGURE 3:** Measurement model. ^***^p < 0.001.

**TABLE 4:** Structural model results effects.

Structural paths	Proposal effect	Estimate	S.E.	*T*-Value	Decision
BAA → IPB	(H1) +	0.246***	0.108	2.277	Supported
BAA → ECBR	(H2) +	0.190***	0.054	3.508	Supported
ECBR → IPB	(H3) +	0.408**	0.143	2.864	Supported
BAA*BC → IPB	(H4) +	0.253**	0.082	3.081	Supported
ECBR*BC → IPB	(H5) +	0.364**	0.072	5.055	Supported

***Significant at the 0.001 level; **significant at the 0.01 level.

**TABLE 5:** Direct, indirect, and total effects analysis.

					Bias-corrected confidence intervals	
	Proposal effect	Direct effects	Indirect	Total	Lower confidence level	Upper confidence level
			effects	effects		
BAA → ECBR → IPB	**(H2a)** +	0.246***	0.051**	0.297***	0.03	0.164

***Significant at the 0.001 level. **significant at the 0.01 level.

#### Direct Effects

The results of path analysis of the aforementioned structural equation model are summarized in Figure 3 and Table 4, and the conclusions of each hypothesis can be obtained. In Table 5, statistically significant (*p*-values), *T-Value*, standard error and path coefficients (β) are presented. These values provide good basis to decide the acceptance or rejection of a hypothesis. The results in Figure 3 and Table 4 show that both direct relationships are statistically significant had support for the positive effects of BAA on IPB and ECBR. The path from BAA to IPB is used as Hypothesis 1. The value of path coefficients (β) and *p*-value of the path from BAA to IPB are 0.246 and <0.001, respectively. The *p*-value is below 0.05 and path coefficient is positive, which is indicating that the BAA has significant impact on IPB. Therefore, Hypothesis 1 is being accepted. Another path was developed to check the impact of BAA on ECBR. Hypothesis 2 was designed to show second relation. The path coefficient and *p*-value for Hypothesis 2 are 0.1190 and <0.001, respectively, which shows that path is statistically significant at 5% level of significance. Similarly, Hypothesis 2 has been supported.

#### Direct, Indirect, and Total Effects

We also have discussed earlier that the study tests indirect relations along with the direct paths. Similarly, to explore the mediating relations, one mediation hypotheses was proposed. The hypothesis was proposed to check the mediation effects of ECBR on BAA and IPB. The estimated results from mediation testing are presented in Table 5. The results for the mediation of ECBR in the impact of BAA on IPB have indicated that the path coefficient and *p*-value are 0.051 and <0.01, respectively. The *p*-value is below 0.05. Hence, Hypothesis 3 has been accepted. It has been already stated and confirmed that BAA has direct positive effect on IPB. Consequently, it can be said that the mediation is partial mediation. Similarly, it can be concluded that ECBR partially mediates the relationship between BAA and IPB.

#### Moderating Effects of Brand Commitment

For H4, to test the moderating effects of Brand Commitment, we added the interactions between BAA and BC in the model. The findings of H4 predicts that the higher the BC, the higher is the effect of BAA on IPB. The results of moderating analysis in Figure 4 and Table 3 reveal a positive and significant interaction effect between BAA and BC on IPB (β = 0.253, *p* < 0.01), which indicates that BC strengthens the positive effects of BAA on IPB. Next for H5, to test the moderating effects of Brand Commitment in the relationship between ECBR and IPB, we added the interactions between ECBR and BC in the model. The findings reveal that the higher the BC, the higher is the effect of ECBR on IPB. The results of moderating analysis in Figure 5 and Table 3 showed a positive and significant interaction effect between ECBR and BC on IPB (β = 0.364, *p* < 0.01), which indicates that BC strengthens the positive effects of ECBR on IPB.

**FIGURE 4:** Moderating effects of BC.

**FIGURE 5:** Moderating effects of BC.

## Discussion and Implications

The purpose of this study was to determine whether brand managers might achieve desired outcomes, such as increasing people’s likelihood to purchase a product from a luxury brand, by strengthening the relationship between brand attribute associations and E-CBRs. The study employed SEM to demonstrate that E-CBR had a significant effect on people’s want to purchase an extension of a luxury brand, as well as a significant effect on the relationship between brand attribute associations and desire to purchase the extension. This study established a link between customers’ attribute associations with a luxury brand and their emotional attachment to that brand which is parallel with the previous study of Ahn et al. (2018) and contradicted with the findings of prior study of Jacob et al. (2020). This synergy is what motivates consumers to purchase the brand’s new items, demonstrating how critical it is to leverage people’s beliefs and knowledge about the brand to help them develop emotional relationships with it. According to Piehler (2018), brand commitment also influences whether individuals want to purchase an extension of a luxury brand and an extension of ECBR.

### Theoretical Implications

Theoretically, this study provides an intensive knowledge of the association that exists between the intent to buy luxury brands’ extension and E-CBR. This study demystifies the impact of brand attributes (uniqueness, prestigious values, and brand image) and relational factors (brand self-identification and brand love) on the intent to buy luxurious brand extensions. According to this study, consumers use salient cognitive memories and schemas associated with luxury brands and emotional bonds formed with brands to decide on whether to buy brand extensions or not. This study focuses on the heart versus mind distinction, which is integral to the research on the relationship between consumers and brands. The heart represents affective and emotional aspects of the brand-customer relationship, while the mind is all about the cognitive dimensions. Both emotional and cognitive aspects influence the intention to buy luxury brand extensions by operating separately and interdependently in formulating purchase behavior (Ahn et al., 2018).

Besides, this study attempted to create an in-depth theoretical interpretation of the interaction amongst emotional consumer-brand relationships and the intention to buy luxury brands’ extension. In that connection, the study develops a new approach to defining the emotional bonds existing between luxury brands and customers. The new concept integrated all relations aspects of brand self-identification, brand passion, brand love and brand attachment (Chen and Qasim, 2021). Besides, this study contributed to the existing limited literature on conceptualization of brand interactions or appraisals of such relationships when determining how they influence brand extensions. This was through assessing how ECBR affects the intent to buy luxury brands’ extensions (Tong et al., 2018). Most importantly, the study contributes to the limited current knowledge on emotional and cognitive connections existing between consumers in China and their preferred luxury brands.

The study generally creates an in-depth perception of the connection between brand attributes and ECBRs. It contributes to the current literature by combining various important emotional and cognitive elements to form one framework. This study also suggests that developing consumer emotions to brands comes from the cognitive relationship’s consumers have in their minds. The study adds on the existing knowledge regarding the significance of establishing and creating intangible brand attributes interactions that transform perceptions to consumer-brand interactions.

Besides this study confirming that brand commitment moderates the interaction between intention to buy luxury brands’ extensions and brand attribute associations, it also acknowledges that perceived fit facilitates the transfer of perceptions and attitudes from the main brand to its extensions. This study’s findings offer specific theoretical implications to categories whereby brand’s hedonic and unique attributes include important advantages of consumption related to luxury brands. According to this study, brand commitment can extend to luxury brand extensions. But this research failed to highlight the moderating effect caused brand commitment when it comes to the relationship between the intent to buy luxury brands’ extensions and ECBR. According to the study, the categorization of brand extensions does not enhance how ECBRs affect the intention to purchase. Therefore, consumers’ emotional bonds with brands influence their intent to buy brand extensions regardless of the existing commitment.

### Managerial Implications

This study provides several crucial managerial implications. It appreciates the significant role displayed by brand attribute associations alongside its impact on ECBRs development. It is fair to conclude that more focus should be directed to showcasing the emotional and hedonic characteristics of a brand to create a lasting emotional bond with customers. Together with strong symbolic attributes, brand image, prestigious and unique qualities, emotional bonds can influence the intent to buy luxury brand extensions (Prados-Pena and Del Barrio-García, 2021). A strong connection between the parent brand and its extensions positively influences the development of an emotional bond with a brand. Customers need to be constantly told about the unique and prestigious factors of a parent company in order to decide whether to buy the brand’s extension or not (Tsai et al., 2020).

Besides, the study provides empirical evidence on the relationship between brand attribute association and ECBR and their impact on the intent to buy luxury brand extensions. In that connection, brand managers need to use strategies that enhance the bond between emotional and cognitive factors customers associate with a particular brand. Luxury brand managers ought to balance emotionality and rationality to create and capitalize on unique associations with customers. For example, these managers must showcase through adverts the exceptional qualities of the brand while providing rational arguments intended to assist customers in deciding on whether to buy luxury brand extensions.

The study also confirmed the influence ECBR has on the intent to buy luxury brand extensions is not reliant on the existing brand commitment. Therefore, brand managers have an opportunity to capitalize on emotional bonds with their customers to bypass the challenges that emanate from unfit or dissimilar brand extensions. So, to reap from the booming luxury market in China, luxury brand managers must consider putting the brands in various categories instead of common or traditional products to create and maintain emotional attachments with consumers in China. From a general perspective, this study provides luxury brand managers with insight about the growing and under-exploited Chinese market. Findings from the current study are relevant luxury brand managers who want to explore this market.

## Limitations and Recommendations

The current research comes with some limitations that can form a basis for further studies. The conceptual framework only focuses on one important variable: the intent to buy luxury brand extensions. There need to be further studies on other pertinent outcomes such as brand loyalty and positive WOM. Besides, the study is only limited to brand commitment to be the moderator. Further studies need to put into consideration other dimensions such product innovation and extension direction. In the sample, most respondents consisted of young luxury brand customers from China. Even though this study highlights several crucial trends in the constantly growing market, future studies need to look at the various cultural contexts and comparison with older generations. The study capitalized on data collected from targeted retailers of luxury brands, specifically those with high status. Therefore, future studies need to also put into consideration the location of the store. Besides, this study capitalized on mock-up extensions in regards to the choice of the brand extensions. In future studies, actual brands may be used, followed by an evaluation of the brand extensions. Lastly, due to the unique luxury brands’ characteristics, the model of research should draw a comparison in a low involvement setting to determine if similar theoretical links will occur and the impact on the intent to buy brand extensions.

## Data Availability Statement

The raw data supporting the conclusions of this article will be made available by the authors, without undue reservation.

## Author Contributions

Both authors listed have made a substantial, direct, and intellectual contribution to the work, and approved it for publication.

## Conflict of Interest

The authors declare that the research was conducted in the absence of any commercial or financial relationships that could be construed as a potential conflict of interest.

## Publisher’s Note

All claims expressed in this article are solely those of the authors and do not necessarily represent those of their affiliated organizations, or those of the publisher, the editors and the reviewers. Any product that may be evaluated in this article, or claim that may be made by its manufacturer, is not guaranteed or endorsed by the publisher.
